The article "Treatment of Fracture of the Calcaneus via Bone Axial X-Ray Image-Based Minimally Invasive Approach" was published in 2022. Journal: Comput Math Methods Med.

# Treatment of Fracture of the Calcaneus via Bone Axial X-Ray Image-Based Minimally Invasive Approach

**DOI:** 10.1155/2022/3012589

**Published:** 2022-07-01

**Authors:** Jie Xiao, Zengfeng Xin, Xiaojun Fu, Jiaqi Huang, Bi Zhang, Haiping Yu

**Affiliations:** ^1^Department of Orthopedics, The Second Affiliated Hospital (Jiande Branch), Zhejiang University School of Medicine, Jiande, Hangzhou, 311600 Zhejiang, China; ^2^Department of Orthopedics, The Second Affiliated Hospital of Zhejiang University School of Medicine, Hangzhou, 311000 Zhejiang, China

## Abstract

To discuss the values of two bone axial X-ray image-based minimally invasive approach surgeries in the diagnosis and treatment of fracture of the calcaneus, 80 patients diagnosed with fracture of the calcaneus by bone axial X-ray examination were selected and divided equally into the minimally invasive longitudinal approach (MILA) group (40 cases) and the sinus tarsal approach (STA) group (40 cases). Besides, the duration of operation, the incidence of complications, the time-to-start weight training, and the American Orthopaedic Foot and Ankle Society (AOFAS) foot function scoring system between the patients in the two groups were compared. The results showed that the duration of operation and incidence of complications among the patients in the MILA group (42.87 ± 5.12 minutes, 20%) were both superior to those among the patients in the STA group (60.43 ± 7.31 minutes, 32.5%). The time-to-start weight training in the MILA group was 5.2 weeks, which was obviously shorter than that in the STA group (5.7 weeks). The difference in AOFAS scores between the two groups was not significant. The walking pavement score in the MILA group (4.2 ± 0.37 points) was slightly higher than that in the STA group (3.3 ± 0.45 points), and the differences demonstrated statistical meaning (*P* < 0.05). To sum up, the bone axial X-ray image is an essential examination method of diagnosing fracture of the calcaneus. The two minimally invasive methods both showed good clinical therapeutic effects. The operation of MILA was relatively shorter with fewer complications and is worthy of being promoted as an effective treatment method of fracture of the calcaneus.

## 1. Introduction

The calcaneus is a very important bone in the foot. When people stand and walk, the calcaneus is needed to support the sole of the foot and is associated with many bones. Calcaneal injuries affect normal function of the foot [1, 2]. Fracture of the calcaneus is a common fracture usually caused by trauma, such as falling from heights, landing on the foot, or vertical force to the heel. Fracture results in the pains and swelling in the heel, shallower posterior sulcus of the ankle, contusion as well as ecchymosis in the ankle of the foot, and even walking difficulty or ankle injury [3–5]. Fracture of the calcaneus caused great pressure on patients and their family members. Hence, patients should receive timely diagnosis and treatment in the hospital once they suffer from the above symptoms. X-ray is the most basic imaging examination method and the basis of guiding the treatment plan for the diagnosis of fracture of the calcaneus, including lateral and axial radiographs [6, 7]. Bohler and Gissane were the main references in lateral radiographs. The former one was used to reflect the height of the calcaneus and the level of joint extrusion, while the latter one can assess the positional relation and the level of displacement of articular surfaces. Axial X-ray is generally utilized as the method of evaluating calcaneal deformity and broadening and can help check the status of the sustentaculum tali [8, 9]. In the imaging examination of the calcaneus, the axial X-ray is an important method of checking fracture and is widely applied in clinical practice.

The patients with the calcaneal articular surface unaffected, inconspicuous displacement, and minor injury can be performed with nonoperative therapy, such as the external fixation with gypsum or special braces. The patients with obvious displacement and fracture affecting articular surfaces need to receive surgical therapy to restore the normal shape of the calcaneus and the integrity of articular surfaces [10]. Traditional surgical therapy is a lateral dilated incision, which fully exposes the fractured sites. In this case, bone soft tissues are removed massively with a large surgical wound and increased incidence of postoperative complications. With the development of medical technology, minimally invasive surgery is popularized in recent years. It can reduce the incidence of postoperative complications and shorten operation and hospitalization time. Hence, it is applied in clinical practice more and more commonly [11]. The minimally invasive longitudinal approach (MILA) and sinus tarsal approach (STA) are two commonly applied surgical methods at present. Nonetheless, whether there were differences in the therapeutic effects and safety of the two surgical methods was still not clear [12].

To conclude, 80 patients with fracture of the calcaneus who were treated and hospitalized in the orthopedic surgery department of our hospital were selected. According to different surgical methods, they were randomly divided equally into the MILA group (40 cases) and the STA group (40 cases). In addition, the rate of repeated treatment, the calculus clearance rate, the duration of operation, the incidence of complications, the time-to-start weight training, and the American Orthopaedic Foot and Ankle Society (AOFAS) foot function scoring system between the patients in the two groups were compared to evaluate the therapeutic effects and safety of different surgical methods in the fracture of the calcaneus comprehensively, which provided data support for the clinical treatment of the fracture of the calcaneus.

## 2. Materials and Methods

### 2.1. Research Objects

A total of 80 patients with the fracture of the calcaneus treated at the hospital and hospitalized between May 2019 and August 2020 were selected and randomly divided into two groups. The patients in the two groups underwent MILA and STA therapies. Among the 80 included patients, there were 64 males and 16 females aged between 18 and 65 with the average of 42.3 ± 2.6. The subjects had agreed to sign informed consent forms, and the research had been approved by the ethics committee of our hospital.

The inclusion criteria are as follows: all patients diagnosed with intra-articular calcaneal fracture via bone axial X-ray imaging examination, patients aged 18 or above, patients without a previous fracture of the calcaneus, and patients with complete clinical information and imaging data.

The exclusion criteria are as follows: patients with other injuries to the ipsilateral limb, patients with severe organ diseases and mental diseases, patients with foot deformity, and patients with poor compliance and who were uncooperative in the experiment.

### 2.2. Calcaneal Axial X-Ray Imaging Examination

The X-ray machine was used to perform calcaneal axial examination for the patients. The patients needed to stand or be seated and stretch out their lower limbs. After that, they were instructed to attach the calcaneus on the affected side to the detector and keep the foot sagittal plane perpendicular to the detector. The toe tip of the affected side was pulled back with a cloth strap until the dorsiflexion of the ankle joint occurred. Next, patients should incline 35° to 45° to the head end. Finally, the film was projected horizontally through the center of the calcaneus.

### 2.3. Surgical Treatment Methods

*MILA group*: the entire procedure of the surgery was performed under the supervision of the X-ray machine. Two Kirschner wires (3.5 mm) were inserted into the calcaneus from the posterior of the calcaneal tuberosity. The needle tip should not go beyond the fracture line. The subtalar articular surface was used as the reduction point for the fracture to be reduced into the normal structural range. Besides, the calcaneus was pushed laterally towards the center to assist in successful reduction. Without any abnormality, a Kirschner wire was used for temporary fixation. After that, a longitudinal approach incision with the length of 3 cm was made lateral to the tendo calcaneus and calcaneus. Next, a periosteal stripper was placed into the incision to remove the periosteum. Then, a blade plate was placed and fixed with screws. After the fixation, the incisions were sutured layer by layer.

*STA group*: an incision with the length of about 4 cm was made at the sinus tarsus, and then, the skin was cut layer by layer without the injury to nerves and muscle tendons. During the surgery, the calcaneofibular ligament was cut to fully expose the subtalar joint. Physiological saline was used to rinse a lot of blood clots. Fracture reduction was performed with the periosteal stripper to restore it to the normal structural range. After that, a Kirschner wire was utilized for temporary fixation. Without any abnormality, a blade plate was placed and fixed with screws. After the fixation, the incisions were sutured layer by layer.

*Postoperative processing*: patients could change medications 24 hours after the surgery to keep the wound dry. After 48 hours, they could perform ankle movement and appropriate exercise. According to their own recovery, patients could start weight-bearing walking exercise about 5 weeks after the surgery. According to their own actual situations, patients could remove the fixed blade plate 1 year after the surgery.

### 2.4. Follow-Up and Observation Indexes

Telephone or outpatient follow-up was performed 3, 6, and 12 months after the surgery. The duration of surgery, the incidence of complications, and the time-to-start postoperative weight training of the patients in the two groups were observed and recorded. After the surgery, the American Orthopaedic Foot and Ankle Society (AOFAS) [13] foot function scoring system was adopted to assess the calcaneal recovery among the included patients. The scores ranging between 90 and 100 points indicated excellent, the scores ranging between 80 and 89 points represented good, the scores ranging between 70 and 79 points meant qualified, and the scores less than 70 points suggested poor.

### 2.5. Statistical Analysis

The statistical analysis of all experimental data was carried out using SPSS 24.0 software. Measurement data were expressed via mean + standard deviation ( x ± s), and enumeration data were denoted by the *χ*^2^ test for statistical inference. Measurement data conformed to normal distribution using the *t* test. *P* < 0.05 indicated statistical meaning.

## 3. Results

### 3.1. Comparison of General Data

According to Figure 1 below, there was no apparent difference except for comparability in age, gender, body mass index (BMI), and fracture Sanders classification of the patients in the two groups (*P* > 0.05).

### 3.2. Case Analysis

A male patient aged 38 in the MILA group was admitted to the hospital with the chief complaint of “left calcaneus comminuted fracture caused by accidentally falling off on bicycle.” Calcaneal axial X-ray examination was performed to observe foot broadening with varus deformity (Figure 2). After the discussion on the disease, left calcaneus MILA surgical treatment was performed.

A male patient aged 64 in the STA group had the chief complaint of “left foot pain for 7 hours after falling from a height.” After the clinical discussion, it was determined that STA surgery was carried out after complete detumescence. Postoperative left calcaneal axial X-ray slice examination was performed to show good para position between the calcaneal tuberous angle and the cross angle and between the anterior articular surface and the posterior articular surface, as shown in Figure 3 below.

### 3.3. Comparison of Operation Time

According to Figure 4, the operation time of the MILA group was 42.87 ± 5.12 minutes, which was significantly shorter than that of the STA group (60.43 ± 7.31 minutes). The differences revealed statistical meaning (*P* < 0.05).

### 3.4. Comparison of Complications

According to Figure 5, there were 2 patients suffering from superficial infection, 1 suffering from deep infection, 2 suffering from gastrocnemius nerve injury, and 3 suffering from plantar nerve injury in the MILA group. The incidence of complications in the MILA group was 20%. In the STA group, there were 2 patients with superficial infection, 2 with deep infection, 1 with skin edge necrosis, 2 with gastrocnemius nerve injury, and 4 with plantar nerve injury. The incidence of complications in the MILA group amounted to 32.5%. The incidence of complications in the MILA group was much lower than that in the STA group, and the difference revealed statistical meaning (*P* < 0.05).

### 3.5. Comparison of Time-to-Start Weight Training

According to Figure 6, weight functional training began after surgery. The time-to-start weight training in the MILA group was 5.2 weeks, which was obviously shorter than that in the STA group (5.7 weeks). The difference suggested statistical meaning (*P* < 0.05).

### 3.6. Comparison of AOFAS Scores between the Two Groups

According to Figure 7, AOFAS scores, including the activity restriction, pain, walking distance, and total scores, in the MILA group and the STA group all showed no significant differences (*P* > 0.05). In terms of walking pavement score, 4.2 ± 0.37 (MILA group) was apparently superior to 3.3 ± 0.45 (STA group). The differences demonstrated statistical difference (*P* < 0.05).

## 4. Discussion

Fracture of the calcaneus is a common fracture usually caused by falling from a height, landing on the heel, and vertical force to the heel. As a result, excessive swelling of the heel, the shallowing of the posterior sulcus of the ankle, and the compression as well as pain of the heel occur [14, 15]. The patients with fracture of the calcaneus with the calcaneal articular surface unaffected and inconspicuous displacement can be performed with nonoperative external fixation [16]. The patients with the injuries to articular surfaces (75% to posterior articular surface and 63% to calcaneocuboid joint surface) need to receive surgical therapy. In most cases, a special internal fixation device is utilized to restore the width and height of the calcaneus, which promotes the recovery of the subtalar articular surface as soon as possible to enable them to get down on the ground for weight training. Nevertheless, traditional open reduction surgery leads to high incidence of complications, which seriously affects the postoperative recovery of patients. The minimally invasive approach technique is widely applied in clinical practice [17, 18].

The experiment was performed on 80 patients with fracture of the calcaneus divided into two groups. According to their calcaneal axial X-ray slices, they were performed with MILA and STA surgeries. Besides, the duration of operation, the incidence of complications, time-to-start weight training, and AOFAS scores in the two groups were observed and comprehensively assessed. The results revealed that the calcaneal axial X-ray slice demonstrated significant reference values in the diagnosis of fracture of the calcaneus. The duration of surgery in the MILA group was relatively shorter with lower incidence of postoperative complications (*P* < 0.05), which was consistent with the study results obtained by Stinton et al. [19]. The incisions made in MILA surgery do not intersect with foot blood vessels and cause little influence on bone blood flow. Consequently, the injury to nerves was minor with a low incidence of postoperative complications.

Clinical practice has confirmed that early initiation of weight-bearing activity after the surgery on fracture of the calcaneus was more beneficial to functional recovery. According to the experimental results, the time-to-start weight training in the MILA group was 5.2 weeks, which was obviously shorter than that in the STA group (5.7 weeks) (*P* < 0.05). The difference indicated that MILA surgery could provide strong fixation of the fractured calcaneus and pain relief. Hence, patients were allowed to perform weight-bearing exercises earlier, which was also mentioned in the article composed by Cao et al. [20]. In terms of the AOFAS score, the experimental results demonstrated that the difference in AOFAS scores between the two minimally invasive approach therapies was not significant. Only the walking pavement score in the MILA group was slightly higher than that in the STA group (*P* < 0.05), which suggested that both MILA and STA showed excellent clinical therapeutic effects and played positive roles in the recovery of patients' calcaneus. Zhan et al. [21] pointed out that STA could expose the articular surface and promote the restoration of its normal smoothness. In contrast, MILA could realize the direct vision of the articular surface, the recovery function of the articular surface could be enhanced, and the time of union of the fracture could be improved by patients' early weight-bearing training. Hence, the clinical therapeutic effects of the two surgical methods were approximately equal.

## 5. Conclusion

In this research, 80 patients diagnosed with fracture of the calcaneus via bone axial X-ray examination were selected and divided equally into the MILA group (40 cases) and the STA group (40 cases). Finally, it was found out that bone axial X-ray imaging could guide the procedure of surgical treatment of fracture of the calcaneus and assess patients' bone recovery. The therapeutic effects of MILA and STA on fracture of the calcaneus were similar. However, the duration of MILA was shorter with fewer postoperative complications. Hence, it was the preferred choice for clinical treatment. Unfortunately, the sample size of included patients was small with a single source. Besides, the AOFAS scoring system has disadvantages in the numerical design though it is widely applied. Hence, a wider range of case data would be included in follow-up studies. The follow-up period would be extended to further discuss the selection of treatment plans for the fracture of the calcaneus. To sum up, the research provided data reference for the clinical diagnosis and treatment of the fracture of the calcaneus.

## Figures and Tables

**Figure 1:** Comparison of general data on the patients in the two groups: (a) comparison of age; (b) comparison of gender; (c) comparison of BMI; (d) comparison of fracture classification.

**Figure 2:** MILA surgery: (a) preoperative left calcaneus axial X-ray slice; (b) postoperative left calcaneus axial X-ray slice.

**Figure 3:** STA surgery: (a) preoperative left calcaneus axial X-ray slice; (b) postoperative left calcaneus axial X-ray slice.

**Figure 4:** Comparison of operation time between the two groups. ^∗^The comparison of operation time between MILA group and STA group, *P* < 0.05.

**Figure 5:** Comparison of the complications between the two groups. (a) Number of complications in the two groups (A represents superficial infection; B denotes deep infection; C refers to skin edge necrosis; D represents gastrocnemius nerve injury; E denotes plantar nerve injury); (b) comparison of the complications between the two groups. ^∗^The comparison of the incidence of complications in the MILA group with the STA group, *P* < 0.05.

**Figure 6:** Comparison of time-to-start weight training between the two groups. ^∗^The comparison of time-to-start weight training in the MILA group with the STA group, *P* < 0.05.

**Figure 7:** Comparison of AOFAS scores between the two groups. (a) Comparison of scores for activity restriction, pain, walking distance, and walking pavement between the two groups; (b) comparison of total AOFAS scores between the two groups. ^∗^The comparison of AOFAS score for walking pavement in the MILA group with the STA group, *P* < 0.05.

## Data Availability

The data used to support the findings of this study are available from the corresponding author upon request.
